# Intelligent Diagnosis of Heart Murmurs in Children with Congenital Heart Disease

**DOI:** 10.1155/2020/9640821

**Published:** 2020-05-09

**Authors:** Jiaming Wang, Tao You, Kang Yi, Yaqin Gong, Qilian Xie, Fei Qu, Bangzhou Wang, Zhaoming He

**Affiliations:** ^1^Research Center of Fluid Machinery Engineering and Technology, Jiangsu University, Zhenjiang, Jiangsu 212013, China; ^2^Department of Cardiovascular Surgery, Gansu Provincial Hospital, Lanzhou, Gansu 730000, China; ^3^Congenital Heart Disease Diagnosis and Treatment, Gansu Province International Science and Technology Cooperation Base, Lanzhou, Gansu 730000, China; ^4^Emergency Center, Children's Hospital of Anhui Province, Hefei, Anhui 230051, China; ^5^Shanghai Lishen Information Technology Co., Ltd., Shanghai 200000, China; ^6^College of Information Science and Technology, Gansu Agricultural University, Lanzhou, Gansu 730070, China; ^7^Department of Mechanical Engineering, Texas Tech University, Lubbock, TX 79409, USA; ^8^Beijing Advanced Innovation Center for Biomedical Engineering, Beihang University, Beijing 100083, China

## Abstract

Heart auscultation is a convenient tool for early diagnosis of heart diseases and is being developed to be an intelligent tool used in online medicine. Currently, there are few studies on intelligent diagnosis of pediatric murmurs due to congenital heart disease (CHD). The purpose of the study was to develop a method of intelligent diagnosis of pediatric CHD murmurs. Phonocardiogram (PCG) signals of 86 children were recorded with 24 children having normal heart sounds and 62 children having CHD murmurs. A segmentation method based on the discrete wavelet transform combined with Hadamard product was implemented to locate the first and the second heart sounds from the PCG signal. Ten features specific to CHD murmurs were extracted as the input of classifier after segmentation. Eighty-six artificial neural network classifiers were composed into a classification system to identify CHD murmurs. The accuracy, sensitivity, and specificity of diagnosis for heart murmurs were 93%, 93.5%, and 91.7%, respectively. In conclusion, a method of intelligent diagnosis of pediatric CHD murmurs is developed successfully and can be used for online screening of CHD in children.

## 1. Introduction

Pulsatile blood flow and tissue motion such as heart valve opening and closing occur in the heart due to myocardial contraction and relaxation. Pressure wave or fluctuation associated with the flow or tissue motion is considered to be the cause of heart sound which travels out to chest wall and is heard with a stethoscope. The heart sound can be recorded by an electronic stethoscope to generate phonocardiogram (PCG) which are acoustic waves. The first (S1) and second (S2) heart sounds are heard and caused by closing of the atrioventricular and semilunar valves, respectively [1, 2], and reflected in PCG as two distinct groups of fluctuation signals. Rarely, the weak third (S3) and forth (S4) heart sounds can be heard which are related to ventricular inflow and atrial contraction, respectively [3]. Normal heart sounds usually contain S1 and S2 only without murmur which is noise between S1 and S2. Heart murmurs usually include pathological murmur, which is caused by abnormal blood jet through the defective heart valves, septum, and narrowing arteries in the heart, and innocent murmur, which is primarily due to physiologic conditions outside the heart. Pathological murmur is associated with heart pathologies which include stenotic or regurgitant heart valves, septal defects, patent foramen ovale, tetralogy of fallot, pulmonary stenosis, and patent ductus arteriosus. Therefore, heart auscultation has been used for diagnosis and monitoring of heart diseases. Intelligent heart auscultation is desired for screening or monitoring of patients with heart diseases and can be developed into a wearable device for Internet medicine.

Accurate detection of heart murmurs from PCG signal is a main task in intelligent auscultation. PCG signal processing includes three major steps: PCG segmentation, feature extraction, and PCG classification. First, PCG segmentation is to locate S1 and S2 from PCG signal. Electrocardiogram signal is applied to assist in the PCG segmentation in early studies [4, 5], but it is not convenient, especially for infants. Empirical mode decomposition [6] can be used to locate S1 and S2 by selecting appropriate intrinsic mode functions, in which end point effect caused by cubic spline interpolation leads to artifacts and distortion of the decomposed PCG signal. The PCG envelope-based [7, 8] and wavelet transform [9–11] are most commonly used for PCG segmentation and are effective in segmentation of mild heart murmurs only. Both methods are limited in moderate and severe heart diseases in which murmurs suppress or overlap with S1 or S2 in both time and frequency domains [12]. Therefore, a segmentation method that can also locate moderate and severe heart murmurs is needed. Meanwhile, the hypothesis that the duration of systole was shorter than that of diastole was valid for adults PCG segmentation [7, 13], but not for children. Children have a fast and widely distributed heart rate and may have a shorter diastole [5]. It is better to decide the systole and diastole based on children's heart rate. Second, the commonly used features in previous studies include magnitude [14], frequency spectrum [10, 15], normalized energy spectrum [16], power spectral density [17, 18], and wavelet coefficients [19]. The differences in these features between heart murmurs and normal heart sounds in both time and frequency domains are used to differentiate heart murmurs from PCG signal. However, the characteristics in the signals other than S1 and S2 in a cardiac cycle are the real key features which differ between the normal heart sounds and heart murmurs. Therefore, selection of time-frequency features from the specific signals as the input of classifier is crucial for classification accuracy. Third, artificial neural network is one of the most commonly used classifiers with very good performance [20, 21] and is adopted usually.

At present, children receive less attention in comparison with adults in PCG studies. The focus of previous pediatric studies is generally distinguishing between innocent murmur [16, 22] or Still's murmur [23] and pathological murmur. Study of prenatal CHD murmur mainly focuses on PCG segmentation but does not involve artificial neutral network diagnosis [24]. The pediatric PCG signal sometimes contains more noises due to movement or crying of children. Furthermore, incidence of CHD in children is high in rural areas of western China. Developing a convenient and low-cost method to screen children in the regions before they are called for an in-hospital check is desirable. Therefore, intelligent diagnosis of pediatric CHD murmurs is challenging and demanding. In this study, a method of intelligent diagnosis for heart murmurs in children with CHD was to be developed.

## 2. Materials and Methods

Figure 1 shows a schematic of normal PCG signal and nomenclature. S1 or S2 was a duration rather than an instant in terms of PCG magnitude. Systole was defined as the duration from the S1 to S2 starting time, and diastole from the S2 to S1 starting time. The closed atrioventricular valve (CAV) and closed semilunar valve (CSV) were the other two durations other than the S1 and S2 durations in a cardiac cycle. S1 and S2 instants were defined to represent instants of the maximal magnitudes of the S1 and S2 durations, respectively.

The flow of PCG processing in this paper was described as follows. First, S1, S2, CAV, and CSV were separated from PCG signal. Then, time-frequency features of CAV and CSV were extracted and fed into an artificial neural network classification system to identify CHD murmur from PCG signal.

### 2.1. PCG Recording

An electronic stethoscope (ChildCare G-100, Shanghai Tuoxiao Intelligent Technology Co., Ltd, Shanghai, China) was used to record PCG signals of 86 pediatric patients aged from 4 months to 16 years, where 24 had normal heart sounds and 62 had CHD murmurs, and digitize PCG signal to 16-bit data at a sampling rate of 44.1 KHz. The PCG signals were recorded at one of five auscultation sites: the aortic valve area, pulmonary valve area, second aortic valve area, tricuspid valve area, and mitral valve area. The recording time of each subject was ∼20 s. The PCG signals were saved in .wav audio format with 8 KHz sampling rate. Patients were from Children's Hospital of Anhui Province, Gansu Provincial Hospital and Health Centers covering eight counties of Qingyang City, Gansu Province. All the subjects have signed the informed consent form with the hospitals. The heart diseases of all the patients were confirmed by the cardiologists in these hospitals according to echocardiography.  Figure 2 shows the pathological distribution of 86 subjects.

### 2.2. PCG Normalization and Denoising

Matlab R2014a (MathWorks, Natick, MA, USA) was used to process the PCG signal. The recorded PCG signal was downsampled by 2 KHz and then normalized to be within ±1.0 to remove differences in the magnitudes among the samples. The normalized PCG signal was denoised by discrete wavelet transform. Daubechies 6 was used as the wavelet basis function and a universal threshold was used in discrete wavelet transform with five decomposition levels. The wavelet coefficients were obtained and processed by a soft threshold function:.

(1) $$\begin{array}{c} W_{\text{new}}=\left\{\begin{array}{cc} \mathrm{sgn}\left(W\right)\left(\left|W\right|-T\right), & \left|W\right|\geq T,\\ 0, & \left|W\right|<T, \end{array}\right. \end{array}$$

where *W* and *W*_new_ are the original and new wavelet coefficients, respectively, and *T* is the universal threshold. The denoised PCG signal was reconstructed by the new wavelet coefficients using inverse discrete wavelet transform [24].

### 2.3. PCG Segmentation

The methods described below were used in order to separate S1, S2, CAV, and CSV from the denoised PCG signal.

#### 2.3.1. PCG Decomposition and Recombination

Figure 3 shows a block diagram of PCG decomposition and recombination. In the PCG decomposition stage, the denoised PCG signal Xd was decomposed into the approximation and detail coefficients by discrete wavelet transform with the Daubechies 6 wavelet basis function and five decomposition levels. The approximation (A1∼A5) and detail (D1∼D5) signals were obtained by reconstructing the coefficients of each level. The Hadamard product of D4 and D5 was performed to obtain the low-frequency recombined signal S which mainly includes S1 and S2. The Hadamard product method is defined as

(2) $$\begin{array}{c} S=\text{D}4.*\text{D}5, \end{array}$$

where *S* is the recombined signal and D4 and D5 are the detail signals of the fourth and fifth levels.

#### 2.3.2. Envelope Extraction

The normalized average Shannon energy was used to extract the envelope of the recombined signal S. A sliding window of 20 ms with a 10 ms overlap was used to calculate the average Shannon energy which is defined as

(3) $$\begin{array}{c} E_{s}=-\frac{1}{N}\sum_{i=1}^{N}s_{\text{norm}}^{2}\left(i\right)\log\;s_{\text{norm}}^{2}\left(i\right), \end{array}$$

where *S*_norm_ is the normalized signal of S with magnitude in ±1.0 and *N* = 40. The normalized average Shannon energy is defined as

(4) $$\begin{array}{c} NE_{s}\left(t\right)=\frac{E_{s}\left(t\right)-M\left(E_{s}\left(t\right)\right)}{S\left(E_{s}\left(t\right)\right)}, \end{array}$$

where *E*_*s*_(*t*) is the average Shannon energy related to the timeline, *M*(*E*_*s*_(*t*)) is the mean value of *E*_*s*_(*t*), and *S*(*E*_*s*_(*t*)) is the standard deviation of *E*_*s*_(*t*).

#### 2.3.3. PCG Components

S1 and S2 instants were determined before S1 and S2 durations in this study. The peaks of the recombined signal S envelope were detected based on the symbol change of the magnitude difference between consecutive sample points in envelope curve. The instants of the peaks were the candidates for S1 and S2 instants. Two constraints on the candidates were applied: (1) only candidates with the maximal magnitude within the range of 100 ms centered on them were reserved, and (2) the time interval between two adjacent candidates was more than 180 ms and less than 500 ms. The filtered candidates were considered to be the S1 or S2 instants. The S1 or S2 instants were used to compute the heart rate as follows:

(5) $$\begin{array}{c} \text{HR}=\frac{60}{1/\left(M-2\right)\sum_{i=1}^{M-2}\left(p_{i+2}-p_{i}\right)}, \end{array}$$

where HR is the heart rate, *M* is the number of S1 or S2 instants, and *p* is the S1 or S2 instant.

It was hypothesized that the duration of systole was shorter than that of diastole at heart rate <= 130 and greater than diastole otherwise. The hypothesis was used to determine S1 and S2 instants. Two time intervals between three consecutive S1 or S2 instants were computed. The shorter one indicated an interval from S1 to S2 instants at heart rate <= 130 or an interval from S2 to S1 instants at a heart rate > 130. Thus, S1 and S2 instants were determined. In order to determine the starting and ending times of S1 and S2 duration, two windows of 120 ms and 100 ms were centered on S1 and S2 instants, respectively. All the envelope data points in the windows with magnitude below 10% of the magnitude of S1 and S2 instants were marked. The boundary data points of the marked points were considered to be boundaries of S1 and S2 duration with the left and right boundaries being the starting and ending times, respectively. Furthermore, CAV and CSV durations were determined from the S1 and S2 boundaries.

### 2.4. Feature Extraction

The maximum (positive), minimum (negative), and the mean absolute values during CAV and CSV were calculated. Their averages based on all the cardiac cycles were used as six time-domain features. The Welch method [25] which had the Hanning window with 50% overlap was used to calculate the power spectral density during CAV and CSV. The maximum and mean values of power spectral density were calculated and their averages based on all cardiac cycles were used as four frequency-domain features. A total of 10 time-frequency features were used.

### 2.5. PCG Classification

The classification system was composed of 86 artificial neural networks with a three-layer network structure in Figure 4 for each one, with 10 neurons in the input layer, 10 neurons in the hidden layer, and one neuron in the output layer. Each artificial neural network takes the 10 extracted features as input and output 0 or 1, corresponding to the normal heart sound and CHD murmur, respectively. The 10 extracted features were normalized to ±1 before training or testing with Neural Network Toolbox in Matlab R2014a. The parameters of artificial neutral network were set as follows: learning rate with an initial value of 0.01, maximum number of iterations of 1000, and target of 10^−6^. Hyperbolic tangent and linear functions were used as activation functions of the hidden layer and output layer, respectively. Levenberg-Marquardt optimization algorithm [26] was used to find the optimal weight parameters of W1 and W2 and the bias of Bias1 and Bias2. Mean squared error loss was used to measure the discrepancy between the predicted value and given output.

The Jack-Knife method [16] was used to evaluate generalization ability of the classification system. This is an iterative process in which one sample was left out each time and used for validation of the classifier which was trained using the other samples. Consequently, 86 artificial neural networks were trained with the 85 samples and validated with the one left-out sample. The above 86 artificial neural networks were combined into a classification system. The predicted value of the classification system was quantified to 0 (≤0.5) or 1 (>0.5) by a threshold of 0.5.

The performance of the classification was evaluated using benchmark metrics such as the accuracy, sensitivity, and specificity, which were defined as

(6) $$\begin{array}{c} \text{Acc}=\frac{\left(\text{TP}+\text{TN}\right)}{\left(\text{TP}+\text{FP}+\text{TN}+\text{FN}\right)},\\ \text{Se}=\frac{\text{TP}}{\left(\text{TP}+\text{FN}\right)},\\ \text{Sp}=\frac{\text{TN}}{\left(\text{TN}+\text{FP}\right)}, \end{array}$$

where Acc is accuracy, Se is sensitivity, Sp is specificity, TP is true positive, FP is false positive, TN is true negative, and FN is false negative.

## 3. Results

### 3.1. PCG Normalization, Denoising, and Segmentation

The baseline in the PCG signal was smoother and the burrs were reduced after denoising which was not shown here.  Figure 5 shows the results of signal recombination and its normalized average Shannon energy for three consecutive cardiac cycles of the PCG signal of a patient with severe VSD. The signal components of S1 and S2 were more prominent than others in the recombined signal, and the low magnitude signals were attenuated more than high amplitude signals in the envelope.

Figure 6 shows the results of PCG segmentation for the same patient with severe VSD. S1 and S2 instants were detected in the envelope, and S1 (the red dotted line), S2 (the blue dotted line), and CAV and CSV in the denoised PCG signal were located.

### 3.2. PCG Feature Extraction

Figure 7 shows the time-frequency distribution of CAV and CSV for the same patient with severe VSD. The magnitude of CAV was more than that of CSV because VSD murmur is one of the systolic murmurs. The overall power spectral density of CAV was greater than that of CSV.

### 3.3. PCG Classification

Figure 8 shows the results of classification for 86 samples with normal heart sounds of #1 to #24 and CHD murmurs of the rest. The false prediction in samples were marked with the red circles. There were two false predictions in normal heart sounds and four false predictions in CHD murmurs. The accuracy, sensitivity, and specificity of diagnosis for heart murmurs were 93%, 93.5%, and 91.7%, respectively.

## 4. Discussion

A method of intelligent diagnosis for heart murmurs in children with CHD was successfully developed. The new segmentation method which utilizes both discrete wavelet transform and the Hadamard product was effective to locate S1 and S2 even in children with moderate and severe CHD diseases whose murmurs suppress S1 or S2. The selected time-frequency features in CAV and CSV durations of PCG signal were closely correlated to CHD murmurs which were associated with pathologies. The traditional classification system based on artificial neural networks worked well in the identification of CHD murmurs. The method promotes development of Internet medicine with heart auscultation devices and intelligent diagnosis of children's CHD.

CHD is the most common heart disease in children, especially in western mountain plateau area with poor medical and transportation conditions. It is the main cause of death in children under five years of age because children in the area often miss the golden period of treatment due to untimely screening. Therefore, there is an urgent need for developing a low-cost screening tool to detect pediatric CHD murmurs. Intelligent auscultation is a solution. The volunteers who are trained to use an electronic stethoscope will go to the less populated region to provide a screening service.

### 4.1. PCG Segmentation

PCG envelope-based or wavelet transform method is a common segmentation method to locate S1 and S2. However, these methods are limited in the segmentation of moderate and severe heart murmurs which often suppress or overlap with S1 or S2 in both time and frequency domains. The PCG envelope-based method separates S1 and S2 from heart murmurs only in time domain. It is impossible to find the peaks of S1 and S2 by a threshold once murmurs suppress S1 or S2. The wavelet transform method separates S1 and S2 by reconstructing low-frequency signals. However, the overlaps of murmurs in time domain cannot be eliminated well by frequency selecting alone, which results in inaccurate location of S1 and S2. In the current study the discrete wavelet transform combined with the Hadamard product was performed to separate murmurs and S1 and S2 in both domains. The low-frequency signals were firstly obtained by the discrete wavelet transform, and then the Hadamard product was performed on the signals to eliminate overlaps in time domain. The results confirmed that the proposed method was suitable for the moderate and severe CHD murmurs.

Another important criteria to decide the systole and diastole in this paper was the hypothesis that the duration of systole is shorter than that of diastole at heart rate<=130. Children have a fast and widely distributed heart rate with inconsistent relationship between the systole and diastole durations. There were a few patients with a heart rate of more than 130 in this study. For example, the heart rate of a 3-month VSD patient was 143, and that of a 5-month PFO patient was 136. The criteria help to avoid displacement of S1 and S2.

### 4.2. PCG Classification

Signals in CAV and CSV are associated with murmurs due to most heart pathologies and should be used as classification features. Time-frequency features in CAV and CSV were extracted in the current study. These features differed from a previous study which extracted features over a whole cardiac cycle even if these features in the current study were similar to those in the previous studies. The current results were excellent because of close association of the features in CAV and CSV with the heart pathologies. These features in CAV and CSV can be further analyzed to indicate specific pathologies in the future. The identification accuracy of CHD murmurs was excellent.

The samples with error classification were checked. One normal heart sound was mistakenly classified as CHD murmur because the noises in the process of PCG recording were classified as murmurs. The noises might be caused by friction during the recording or by children moving and crying and were not removed by the denoising process. The other samples which classified the CHD murmurs as the normal heart sound were four patients. Two of them had mild atrial septal defect and the other two patients had mild ventricular septal defect. These heart murmurs were so weak that the features were close to the normal heart sound.

### 4.3. Performance Comparison

The performance of the current method was compared with those of the previous studies in pediatric PCG segmentation or classification, as shown in Table 1. Performance of the methods in all the studies was above 90% except in the fourth study [24]. The current method had the best accuracy and sensitivity but had low specificity, which indicated that the current method was capable of accurate detection of CHD murmurs but might increase the probability of false positives. In general, the current method had comparable performance in diagnosis of CHD murmurs.

### 4.4. Limitations

The denoising method used in this paper was not able to remove strong noises coming from children crying and moving during the recording. The output data in the prediction were volatile because the mild, moderate, and severe murmurs were not graded. The sample size was relatively low. The PCG signals were recorded at one of five auscultation sites by a professional. The method may not work well if a nonprofessional volunteer records PCG signal by placing an electronic stethoscope in any other position.

## 5. Conclusions

A method of intelligent diagnosis for heart murmurs in children with CHD is successfully developed. The proposed segmentation method is effective in locating S1 and S2 from pediatric CHD murmurs. The selected 10 time-frequency features of PCG signal in CAV and CSV are closely correlated to CHD murmurs. The classification system based on artificial neural networks has a high accuracy in the identification of CHD murmurs. The method promotes development of Internet medicine with heart auscultation devices and intelligent diagnosis of children's CHD.

## Figures and Tables

**Figure 1:** Schematic of normal PCG signal and nomenclature.

**Figure 2:** Pathological distribution of 86 subjects with normal heart sound (normal), ventricular septal defect (VSD), atrial septal defect (ASD), patent foramen ovale (PFO), patent ductus arteriosus (PDA), double outlet right ventricle (DORV), and endocardial cushion defect (ECD).

**Figure 3:** Block diagram of PCG decomposition and recombination.

**Figure 4:** The structure of artificial neural network.

**Figure 5:** The recombined signal and its normalized average Shannon energy.

**Figure 6:** The result of PCG segmentation.

**Figure 7:** The time-frequency distribution of CAV and CSV in cycle #1, 2, 3. (a) The CAV and CSV signal. (b) The power spectral density of CAV and CSV.

**Figure 8:** The result of PCG classification.

**Table 1:** Performance of the current and previous methods in pediatric PCG segmentation or classification.

Method	Segmentation or classification type	Performance
Wavelet transform, singular value decomposition [11]	S1 and S2	Acc = 92.1%
Hilbert envelope, ANN [15]	Normal and six pathologies	Se = 91%, Sp = 94%
Matched filters, support vector machine, ANN [23]	Innocent Still's murmur and other murmurs	Se = 84%∼93% Sp = 91%∼99%
Shannon energy, wavelet transform [24]	S1 and S2	Acc = 88%
Current method	S1, S2, CAV, CSV, normal, and CHD	Acc = 93%, Se = 93.5%, Sp = 91.7%
